The article "Seven-Gene Signature Based on Glycolysis Is Closely Related to the Prognosis and Tumor Immune Infiltration of Patients With Gastric Cancer" was retracted in 2024. Reasons: contaminated cell lines or tissues; unreliable results or conclusions; concerns about the data.

# Seven-Gene Signature Based on Glycolysis Is Closely Related to the Prognosis and Tumor Immune Infiltration of Patients With Gastric Cancer

**DOI:** 10.3389/fonc.2020.01778

**Published:** 2020-09-18

**Authors:** Shanshan Yu, Chuan Hu, Luya Cai, Xuedan Du, Fan Lin, Qiongjie Yu, Lixiao Liu, Cheng Zhang, Xuan Liu, Wenfeng Li, Yu Zhan

**Affiliations:** ^1^Department of Chemoradiation Oncology, The First Affiliated Hospital of Wenzhou Medical University, Wenzhou, China; ^2^Department of Orthopaedic Surgery, The Affiliated Hospital of Qingdao University, Qingdao, China; ^3^Department of Obstetrics and Gynecology, The First Affiliated Hospital of Wenzhou Medical University, Wenzhou, China; ^4^Department of Dermatology, The First Affiliated Hospital of Wenzhou Medical University, Wenzhou, China; ^5^Department of Ultrasound, The First Affiliated Hospital of Wenzhou Medical University, Wenzhou, China

**Keywords:** gastric cancer, glycolysis, prognostic, risk, immune signatures

## Abstract

**Background:** Gastric cancer (GC) is one of the most common malignancies worldwide, exhibiting a high morbidity, and mortality. As the various treatment methods for gastric cancer are limited by disadvantages, many efforts to improve the efficacy of these treatments are being taken. Metabolic recombination is an important characteristic of cancer and has gradually caused a recent upsurge in research. However, systematic analysis of the interaction between glycolysis and GC patient prognosis and its potential associations with immune infiltration is lacking but urgently needed.

**Methods:** We obtained the gene expression data and clinical materials of GC derived from The Cancer Genome Atlas (TCGA) dataset. Univariate and multivariate Cox proportional regression analyses were performed to select the optimal prognosis-related genes for subsequent modeling. We then validated our data in the GEO database and further verified the gene expression using the Oncomine database and PCR experiments. Besides, Gene set variation analysis (GSVA) analysis was employed to further explore the differences in activation status of biological pathways between the high and low risk groups. Furthermore, a nomogram was adopted to predict the individualized survival rate of GC patients. Finally, a violin plot and a TIMMER analysis were performed to analyse the characteristics of immune infiltration in the microenvironment.

**Results:** A seven-gene signature, including STC1, CLDN9, EFNA3, ZBTB7A, NT5E, NUP50, and CXCR4, was established. Based on this seven-gene signature, the patients in the training set and testing sets could be divided into high-risk and low-risk groups. In addition, a nomogram based on risk and age showed good calibration and moderate discrimination. The results proved that the seven-gene signature had a strong capacity to predict the GC patient prognosis. Collectively, the violin plot and TIMMER analysis demonstrated that an immunosuppressive tumor microenvironment caused by hyperglycolysis led to poor prognosis.

The article "Seven-Gene Signature Based on Glycolysis Is Closely Related to the Prognosis and Tumor Immune Infiltration of Patients With Gastric Cancer" was retracted in 2024. Reasons: contaminated cell lines or tissues; unreliable results or conclusions; concerns about the data.

**Conclusion:** Taken together, these results established a genetic signature for gastric cancer based on glycolysis, which has reference significance for the in-depth study of the metabolic mechanism of gastric cancer and the exploration of new clinical treatment strategies.

## Introduction

Gastric cancer (GC) is the fifth most common cancer and the third leading cause of cancer death worldwide (1), seriously threatening human health and causing a heavy blow to the social economy. East Asia, which includes Japan and South Korea, has a significantly higher incidence, with incidence rates that are 2-fold higher in men than in women, according to the GLOBOCAN 2018 estimates of cancer incidence and mortality (1). Most of the patients with GC were in the late stage or local late stage at the time of detection because of occult onset and delayed diagnosis, leading to poor outcomes (2, 3). At present, the clinical comprehensive treatment effect of surgery, radiotherapy and chemotherapy is not ideal, and first-line chemotherapy with platinum-containing drugs in advanced gastric cancer has reached a bottleneck of efficacy (4, 5). Although the development of molecular targeted therapies, such as human epidermal growth factor receptor 2 (HER2) monoclonal antibody, improves the prognosis of advanced gastric cancer, the applicable population is narrow, facing the problem of drug resistance (6–8). Fortunately, many studies have shown that PD-1/PD-L1 immune checkpoint inhibitors have definite efficacy in advanced gastric cancer, which has opened a new avenue for the treatment of gastric cancer (9, 10). However, some GC patients still have poor efficacy (9, 10). Previous studies have reported that some genetic or genomic biomarkers are related to the prognosis of patients with gastric cancer, such as defective DNA mismatch repair (dMMR) (11) and long non-coding RNA (lncRNA) (12–14). Nevertheless, a single gene marker cannot produce good prediction results. Some studies have found that the assessment of genetic traits involving multiple genes can improve the outcome of prognostic prediction (15–17). Therefore, more endeavors are needed to explore more GC biomarkers with high efficiency and sensitivity.

Previous studies have found that the tumor microenvironment significantly affects the diagnosis, survival outcome and clinical treatment sensitivity of patients with gastrointestinal tumors (18, 19). Therefore, evaluating the interactions between tumor cells and the tumor microenvironment may be a new way to find better GC biomarkers. The phenomenon of tumor metabolic reprogramming is widespread, but the root cause of its occurrence is still unknown (20). To adapt to the complex and changeable microenvironment, tumor cells have developed dynamic metabolic heterogeneity, which has become an important feature of cancer (21, 22). One of the most common metabolic reprogramming methods is aerobic glycolysis, of which the Warburg effect is most remarkable. The Warburg effect is a metabolic feature of almost all cancer cells that overconverts glucose into lactic acid, even in the presence of oxygen (23, 24), leading to an acidic environment. As shown in the present study, the inhibition of the tumor glycolysis pathway can effectively inhibit the proliferation of tumor cells and can even play a role in killing tumor cells (25–27). In addition, some glycolytic enzymes have also been proved to be related to the prognosis of GC. Enolase 1 (ENO1) is a metalloenzyme that catalyzes the dehydration of 2-phospho-D-glycerate into phosphoenolpyruvate I during glycolysis, whose ectopic overexpression promotes tumor formation or enhances epithelial–mesenchymal transition (EMT) in gastric cancer (28, 29). The increased level of pyruvate kinase M2 (PKM2), a key enzyme that promotes aerobic glycolysis, is associated with poor survival of GC patients (30). Glucose-6-phosphate isomerase (GPI) is a glycolysis-related enzyme, also known as autocrine motility factor (AMF), which participates in the occurrence of gastric cancer, promotes the invasive phenotype of GC cells, and has a positive correlation with high TNM stage and poor prognosis (31). In short, tumor aerobic glycolysis may be crucial in determining the prognosis and tumor treatment of GC patients. What is more interesting is that the tumor microenvironment (TME) is considered to be a hotbed of tumor cells and is composed of tumor cells, endothelial cells, stromal cells and immune cells, among other cell types (32). This complex process usually contains cellular metabolites, mainly caused by aerobic glycolysis, which is not only a component of energy supply but also plays a role in signal communication between different cells (33). Combined with various complex factors, this will result in the dual characteristics of the immune cells recruited to the tumor site, which plays a pivotal role in the composition and distribution of the tumor immune microenvironment (34). Therefore, searching for more sensitive biomarkers from the perspective of glycolysis is a promising strategy.

The article "Seven-Gene Signature Based on Glycolysis Is Closely Related to the Prognosis and Tumor Immune Infiltration of Patients With Gastric Cancer" was retracted in 2024. Reasons: contaminated cell lines or tissues; unreliable results or conclusions; concerns about the data.

Several research studies have focused on the systematic analysis of glycolysis and tumors, including glioblastoma (15), liver cancer (16), and endometrial cancer (17). However, comprehensive analysis of the interrelation between glycolysis, immune infiltration, and clinical prognosis in GC patients is lacking. In our study, we developed a glycolysis-related signature related to survival on the basis of the gene expression data and clinical materials obtained from The Cancer Genome Atlas (TCGA) GC cohort, which was validated simultaneously in the GEO database. Furthermore, other bioinformatic and statistical methods were adopted to depict the landscape of tumor glycolysis and immunity in gastric cancer, which may bring new insights into the treatment of gastric cancer and the development of new drugs.

## Materials and Methods

### Data Curation Process

Corresponding gene expression data were downloaded from the TCGA database and the GEO database. The RNA sequencing data of 375 GC patients were obtained from the TCGA database and set as the training set, whereas other RNA sequencing data from GSE26253 (*n* = 394), GSE26901 (*n* = 109), GSE66229 (*n* = 300) were downloaded from the GEO database and regarded as testing sets. We also set the exclusion criteria as OS <1 month for research accuracy. As a consequence, we included a total of 1,140 patients for analysis, including 337 patients from TCGA and 803 patients from GEO. Additionally, the complete clinical and survival information of all patients was obtained from TCGA for further analysis.

### Data Processing and Risk Score Calculation

We searched all glycolysis-related gene sets on the Molecular Signatures Database v4.0, comprising five different gene sets (BIOCARTA_GLYCOLYSIS_PATHWAY, GO_GLYCOLYTIC_PROCESS,HALLMARK_GLYCOLYSIS,KE GG_GLYCOLYSIS_GLUCONEOGENESIS, REACTOME_GLY COLYSIS). We ultimately screened out 326 glycolysis-related genes (GRGs) from 56,639 RNA expression profiles as a cornerstone for subsequent research, presented in a Venn diagram. Moreover, gene interaction networks were constructed by inputting these 326 GRGs into Cytoscape and Reactome FI (version 3.7.1); importantly, hub genes were included. We next adopted univariate Cox regression analysis to identify overall survival (OS)-related GRGs. On the basis of univariate Cox regression analysis, we wanted to further define the similarities and differences in the microcosmic characterization of the target glycolytic genes. Circos plots are a powerful visualization tool, with multilayer highly informative circles, suitable for the comprehensive analysis of different genetic information states (35). Therefore, a Circos plot was applied using R language. Then, we applied a least absolute shrinkage and selection operator (LASSO) regression to identify the final elimination of potential predictors with nonzero coefficients (36), which can avoid model overfitting, to select the optimal OS-related GRGs. Afterwards, multivariate Cox regression was carried out to determine the hub genes involved in the final modeling and to obtain a correlation coefficient. The selected mRNAs were divided into risk (hazard ratio (HR) > 1) and protective (0 < HR <1) types. Finally, we constructed a prognostic risk score formula on the basis of a linear combination of the expression levels weighted with the corresponding regression coefficients derived from multivariate Cox analysis. The formula was as follows: Risk score = ∑(β_*n*_ × expression of gene *n*), where β is the regression coefficient.

The article "Seven-Gene Signature Based on Glycolysis Is Closely Related to the Prognosis and Tumor Immune Infiltration of Patients With Gastric Cancer" was retracted in 2024. Reasons: contaminated cell lines or tissues; unreliable results or conclusions; concerns about the data.

### Construction and Verification of the Prediction Model

The data from the TCGA database were employed as the training set as mentioned above. We classified 377 patients with GC from TCGA into two subgroups (high- and low-risk groups) on the basis of the median risk score as the cutoff, and Kaplan–Meier survival analysis was plotted to explore the significant differences in patient survival with the log-rank test. Furthermore, receiver operating characteristic (ROC) curves of 3, 4, and 5 years in R software were generated to calculate the area under the curve (AUC) value of the ROC curve for each predictor model for the purpose of further assessing the efficiency and accuracy of the model. In the test group, namely, data derived from GEO, the same processes were performed to validate the prognostic model of this group. *P* < 0.05 was considered to indicate statistical significance.

### GSVA Between the High- and Low-Risk Group in the Training Set

To further explore the differences in activation status of biological pathways between the high- and low-risk groups in the training cohort, GSVA enrichment analysis was employed by using “GSVA” R packages. GSVA is commonly applied for estimating the variation in pathway and biological process activity in the samples of an expression dataset in a non-parametric and unsupervised method (37). The gene sets of “c2.cp.kegg.v6.2.-symbols” were downloaded from MSigDB database for GSVA analysis. Adjusted P with value less than 0.05 was considered as statistically significance.

### Development of a Nomogram Based on Glycolysis and Clinical Factors

There is a common consensus that the nomogram is a practical tool for clinical application. Therefore, we constructed a nomogram that took glycolysis and clinical variables into consideration using the rms R package. Detailed clinical information of 337 patients with gastric cancer in the training set was shown in Supplementary Table 1. We applied univariate and multivariate Cox regression analyses to identify corresponding variables related to prognosis. Consequently, variables involved in the final nomogram were identified by a backward stepwise variable selection with the Akaike information criterion (AIC). Finally, we created calibration curves to assess the predictive accuracy of the eventual nomogram and adopted the concordance index (C-index) as an index to quantify its discrimination capacity with the help of the Hmisc package (version 4.1.1).

The article "Seven-Gene Signature Based on Glycolysis Is Closely Related to the Prognosis and Tumor Immune Infiltration of Patients With Gastric Cancer" was retracted in 2024. Reasons: contaminated cell lines or tissues; unreliable results or conclusions; concerns about the data.

### Display of the Differential Expression of Hub Genes in the Oncomine Database

To further validate the adverse effects of seven GRGs on tumor development, we utilized the Oncomine database to identify the genes' differential expression between normal tissues and tumor tissues. In this section, we selected *P* < 0.05 or less as a threshold.

### Cell Culture

The human gastric cancer SGC7901, MGC803 and BGC803 cell lines and the normal human gastric epithelial cell line (GES-1) were purchased from Shanghai Cell Bank of the Chinese Academy of Sciences (Shanghai, China). All cells were cultured in PRIM 1640 medium (HyClone, USA) with 10% fetal bovine serum(FBS) and 1% penicillin-streptomycin at a humidified incubator at 37°C with 5% CO_2_. Cells were digested and passaged at a ratio of 1:3 when reaching 90% confluence. Logarithmic growth phase cells were applied for subsequent experiments.

### RNA Extraction and qRT-PCR

We extracted total RNA from the human gastric cancer cells and the normal human gastric epithelial cell employing TRIzol reagent (Thermo Fisher Scientific, Waltham, MA, USA). One microgram of total RNA for the synthesis of single-stranded cDNA was prepared with the help of the PrimeScript RT reagent Kit with gDNA Eraser (Takara Biotechnology Co. Ltd., Dalian, China). Then, we applied reverse transcription quantitative PCR to analyze the expression levels of mRNA of hub genes using a 7,500 PCR system (Thermo Fisher Scientific). The cycling conditions were as follows: 95 minutes or five minutes, followed by 40 cycles of 95°C for 20 s and 60°C for 30 s. The qRT-PCR was operated in triplicate in a 10-μL reaction volume for each sample, and the relative expression levels of STC1, CLDN9, EFNA3, ZBTB7A, NT5E, NUP50, CXCR4 mRNA were calculated by the 2-Ct method. The primer sequences are shown in Supplementary Table 2.

### Exploration of the Immune Infiltration Based on the Seven-Gene Signature

To determine whether and how GRGs affected the tumor-immune microenvironment, a violin plot was constructed to present the contribution of immune cell infiltrations in the high- and low-risk groups using the Fluidigm Singular Analysis Toolset 3.5.2 R package. The tumor immune estimation resource (TIMER) is commonly used to comprehensively analyze the profiles of tumor infiltrating immune cells (38). We employed this software to create corresponding scatterplots and to generate the Spearman correlation, which can be regulated by age or tumor purity (the proportion of cancer cells in the admixture), with the intention of mining the potential relevance of the seven-gene signature on immune infiltration levels.

The article "Seven-Gene Signature Based on Glycolysis Is Closely Related to the Prognosis and Tumor Immune Infiltration of Patients With Gastric Cancer" was retracted in 2024. Reasons: contaminated cell lines or tissues; unreliable results or conclusions; concerns about the data.

### Statistical Analysis

All statistical analyses were performed in R software (version 3.6.1) and GraphPad Prism 7 software. All statistical tests with *P* < 0.05 (two-sided) were statistically significant.

## Results

### Overview of Glycolysis-Related Genes in the TCGA-STAD Cohort

The detailed flow chart of the study design is displayed in Figure 1. In general, we collected and integrated 56,639 RNA expression profiles from 337 GC patients included in the TCGA dataset. We picked out 326 corresponding GRGs for further investigation without differential analysis as a result of the small number of target genes (Figure 2A). To research reciprocal actions among these GRGs, we put the 326 GRGs into Cytoscape to create gene-gene interaction networks (Figure 2B). Cancer-associated proteins, such as GPI (glucose-6-phosphate isomerase), PKG1 (phosphoglycerate kinase 1) and HK (hexokinase), were identified to be major hubs in the resulting networks, which had previously been reported for their association with tumorigenesis (39–41).

**Figure 1:** Flow chart of the systematic identification and comprehensive validation of the seven GRG signature in GC. GC, gastric cancer; TCGA, The Cancer Genome Atlas; GSE, Gene Expression Omnibus Series; OS, overall survival; GRGs, glycolysis-related genes.

**Figure 2:** Overview of glycolysis-related genes (GRGs) in the TCGA GC training cohort. **(A)** Venn diagram showing that glycolysis-related genes belonged to a subset of the whole RNA sequencing of GC in the TCGA dataset. **(B)** Network of glycolysis-related genes in GC constructed by Cytoscape.

### Identification of Survival-Related GRGs in GC

To explore the possible relationship between GRGs and OS in patients with GC, we employed univariate Cox analysis to select survival-related GRGs as preliminary screening in the training cohort. A total of 12 RGRs associated with OS were identified (*P* < 0.05) and are shown in Table 1 with information for gene symbol, HR, 95% CI and *P* value. To check and visualize the status of GRGs, a Circos plot was constructed (Figure 3A) before modeling continued. The locations of all 326 GRGs on the 26 human chromosomes were identified and set in the outermost track. Next, the construction of the middle layer was based on the HR values collected from the univariate Cox regression analysis. In addition, 12 OS-related GRGs were identified and displayed, as illustrated in Table 1. The internal sector was the PPI network, similar to Figure 2B. The medium confidence of the minimum required interaction score was 0.9: specifically, 0.9–0.99 was blue, and >0.99 was red. LASSO regression was next performed to select the optimal OS-related GRGs with nonzero coefficients (Figures 3B,C). We also adopted multivariate Cox regression analysis to further confirm the correlation between these OS-related GRGs and patient survival, finalizing the most significant GRGs involved in the modeling by the stepwise elimination method and obtaining corresponding coefficients. Seven genes (STC1, CLDN9, EFNA3, ZBTB7A, NT5E, NUP50, CXCR4) were identified, as shown in Table 2. These selected genes were separated into the risky type (STC1, CLDN9, NT5E, CXCR4), with HR>1 related to poorer prognosis, and the protective type (EFNA3, ZBTB7A, NUP50), with HR <1 related to better prognosis (Table 2), among which five genes (STC1, CLDN9, ZBTB7A, NT5E, CXCR4) were also considered as independent prognostic factors of GC. Interestingly, ZBTB7A was the only gene that belonged to both protective type and independent prognostic factor, whereas all risk types were independent prognostic factors.

The article "Seven-Gene Signature Based on Glycolysis Is Closely Related to the Prognosis and Tumor Immune Infiltration of Patients With Gastric Cancer" was retracted in 2024. Reasons: contaminated cell lines or tissues; unreliable results or conclusions; concerns about the data.

**Table 1:** Screening GRGs related to survival by univariate analysis in GC patients of the TCGA dataset.

**Gene symbol**	**Overall survival**			
	**HR**	**95.0% CI**		***P***
STC1	1.289	1.097	1.516	0.002
SDC2	1.323	1.105	1.583	0.002
CLDN9	1.240	1.064	1.446	0.006
EFNA3	0.838	0.735	0.954	0.008
SLC35A3	0.716	0.564	0.909	0.006
ZBTB7A	0.632	0.470	0.848	0.002
VCAN	1.271	1.098	1.471	0.001
NT5E	1.295	1.116	1.504	0.001
PLOD2	1.375	1.125	1.679	0.002
NUP50	0.615	0.426	0.887	0.009
GPC3	1.135	1.049	1.228	0.002
CXCR4	1.230	1.077	1.405	0.002

*GRGs, glycolysis-related genes; GC, gastric cancer; TCGA, The Cancer Genome Atlas;HR, hazard ratio*.

**Figure 3:** Circos plot and the least absolute shrinkage and selection operator (LASSO) Cox regression analysis for construction of the final prediction model. **(A)** Circos analysis of glycolysis-related genes from the TCGA whole RNA sequencing. The outermost layer displays the locations of all 326 glycolysis-related genes on the 23 human chromosomes. The middle layer shows the HR values derived from the univariate Cox regression analysis, thus identifying 12 OS-related GRGs, which were illustrated in Table 1. The inner layer shows the PPI network, similar to Figure 2B, whose medium confidence of minimum required interaction score is 0.9, <0.99 is blue, and >0.99 is red. **(B)** Selection of the optimal parameter (lambda) in the LASSO model; dotted vertical lines were drawn at the optimal values by using the minimum criteria. **(C)** LASSO coefficient profiles of the candidate OS-related GRGs with nonzero coefficients determined by the optimal lambda. A coefficient profile plot was produced against the logλ sequence.

The article "Seven-Gene Signature Based on Glycolysis Is Closely Related to the Prognosis and Tumor Immune Infiltration of Patients With Gastric Cancer" was retracted in 2024. Reasons: contaminated cell lines or tissues; unreliable results or conclusions; concerns about the data.

**Table 2:** Identification of the specific seven-GRG signature involved in the establishment of the final prognostic model by multivariate analysis.

**Gene symbol**	**Overall survival**				
	**coef**	**HR**	**95.0% CI**		***P***
STC1	0.170	1.185	1.001	1.403	0.049
CLDN9	0.215	1.240	1.064	1.445	0.006
EFNA3	−0.111	0.895	0.771	1.039	0.146
ZBTB7A	−0.546	0.579	0.420	0.798	0.001
NT5E	0.234	1.263	1.078	1.481	0.004
NUP50	−0.374	0.688	0.460	1.030	0.069
CXCR4	0.166	1.181	1.011	1.378	0.035

*GRGs, glycolysis-related genes; coef, coefficient; HR, hazard ratio*.

### Establishment and Validation of the Seven-Gene Signature for Predicting GC Patient Survival

We established a final prognostic model based on the results of the multivariate Cox regression to more intuitively explore the relationship between the seven GRGs and prognosis. The prognostic risk score formula was specifically constructed according to a linear combination of the expression levels weighted with the regression coefficients from the multivariate Cox regression analysis: Risk score = 0.170 × expression of STC1+0.215 × expression of CLDN9-0.111 × expression of EFNA3-0.546 × expression of ZBTB7A+0.234 × expression of NT5E-0.374 × expression of NUP50 + 0.166 × expression of CXCR4. We then calculated the scores and split the patients into high- and low-risk groups by the median risk score in the training set (Figure 4A). The relationships between survival status and survival times of GC patients ranked by risk scores are shown in Figure 4B. In addition, a heatmap was plotted to show the expression profiles of seven genes (Figure 4C). The expression levels of risky types (STC1, CLDN9, NT5E, CXCR4) were higher in the high-risk group compared to the low-risk group. Conversely, the expression levels of protective types (EFNA3, ZBTB7A, NUP50) were lower in the high-risk group than in the low-risk group, which implied the capacity of the seven-gene signature to accurately predict patient prognosis and their potential impact on the occurrence and development of tumors. The results of Kaplan–Meier survival analysis shed light on the fact that the prediction model possessed powerful capacity to predict the prognosis of GC patients between the low- and high-risk group, in which the low-risk group had a better survival rate than the high-risk group (*P* < 0.0001) (Figure 5A). We then applied the 3-, 4-, and 5-year ROC curves to verify the predictive capacity of the prognostic model; the AUCs of the ROC were almost all ~0.7, suggesting a satisfactory predictive performance (Figure 5B).

The article "Seven-Gene Signature Based on Glycolysis Is Closely Related to the Prognosis and Tumor Immune Infiltration of Patients With Gastric Cancer" was retracted in 2024. Reasons: contaminated cell lines or tissues; unreliable results or conclusions; concerns about the data.

**Figure 4:** Risk score analyses of GC patients in the training cohort based on the seven-GRGs signature. **(A)** Distribution of risk scores per patient. **(B)** Relationships between survival status and survival times of GC patients ranked by risk score. The black dotted line represents the optimum cut-off point dividing patients into low- and high-risk groups. **(C)** Heatmap of the seven-GRG expression profile. Colors from yellow to blue indicate decreasing expression level from high to low.

**Figure 5:** Assessment of the prognostic value of the predictive model in the TCGA GC training cohort. **(A)** Survival analysis of the predictive model. The upper part shows the Kaplan-Meier curves for the high- and low-risk groups; the middle shows the number of living patient variations with time in the high- and low-risk groups; the bottom shows the number of censoring variations with time in the high- and low-risk groups. Red color represents low-risk group data, whereas blue color represents high-risk group data. **(B)** ROC curves of predictive models at 3, 4, and 5 years. Red color represents 3 years, green color represents 4 years, and blue color represents 5 years.

We next validated our seven-gene signature in the testing groups derived from the GEO database to confirm our findings by employing the same model in the training cohort. The patients from GSE26253 (*n* = 394), GSE26901 (*n* = 109), GSE66229 (*n* = 300) were divided into high- and low-risk subgroups by median risk score (Figures 6A,D,G). Consequently, the outcomes of the KM survival curves revealed that the low-risk group had a better survival rate than the high-risk group (Figures 6B,E,H), consistent with the results of the training group. Moreover, we also plotted the 3-, 4-, and 5-year ROC curves to evaluate the predictive efficiencies of the models. The models based on the seven-gene signature demonstrated good sensitivity and specificity, with various AUC values ranging from 0.562 to 0.646 (Figures 6C,F,I).

**Figure 6:** External validation of the prediction model using expression data from the GEO database as testing sets. Patients with low risk scores indicated better OS than those with high risk scores in **(A–C)** GSE26253, **(D–F)** GSE26901, and **(G–I)** GSE66229, which were the same as the results of the TCGA training cohort, suggesting the robust predictive capacity of the prediction model.

The article "Seven-Gene Signature Based on Glycolysis Is Closely Related to the Prognosis and Tumor Immune Infiltration of Patients With Gastric Cancer" was retracted in 2024. Reasons: contaminated cell lines or tissues; unreliable results or conclusions; concerns about the data.

### The Differential Biological Behaviors in High- and Low-Risk Subgroups Identified by GSVA Analysis

Inspired by the satisified ability of the seven-gene signature to predict prognosis in training set and verification set, we further conducted GSVA analysis in order to explore the difference of biological pathway activation state between high- and low-risk groups, with the aim of finding a more comprehensive explanation for prognostic differences between high- and low-risk groups (Figure 7). The heatmap was used to visualize the top 20 biological processes with significant differences ranked from small to large according to P value. We found that the activation pathways of carcinogenesis in high-risk group were significantly enriched, such as gap junction, MAPK signaling pathways, TGF beta signaling pathway, Wnt signaling pathway, etc. This may provide a certain angle of reason for the poor prognosis of the high-risk group.

**Figure 7:** Exploration of the differences of biological behaviors between high- and low-risk groups in training set via GSVA enrichment analysis. The heatmap was used to visualize the top 20 biological processes with significant differences ranked from small to large according to P value, and red represented activated pathways and green represented inhibited pathways.

### Development of a Glycolysis-Clinical Nomogram to Predict the Individual Outcomes of GC Patients

Inspired by the results of the training and testing cohorts, a nomogram was delineated to further predict the individual survival rate of each patient on the basis of glycolysis and clinical factors. First, univariate and multivariate Cox proportional hazard regression models were employed to analyze risk scores and other clinical parameters as covariates. The results of the univariate Cox results revealed that age, stage (T, N, M) and risk were OS-related factors (Figure 8A). Then, with the forward stepwise selection on optimizing AIC applied based on multivariate Cox analysis (Figure 8B), we ultimately chose two variables, including risk and age, for developing subsequent nomograms, which showed that the higher the total score, the shorter the survival time (Figure 9A). There was nice agreement between the predicted value and the actual value, which was confirmed by the calibration curve of the nomogram for the survival probability at 1, 2, or 3 years (Figures 9B–D). We then counted the C-index of the OS nomogram, with the result of 0.651 (95% CI, 0.600–0.702), which suggested greater clinical application value in predicting the long-term survival probability of GC patients.

The article "Seven-Gene Signature Based on Glycolysis Is Closely Related to the Prognosis and Tumor Immune Infiltration of Patients With Gastric Cancer" was retracted in 2024. Reasons: contaminated cell lines or tissues; unreliable results or conclusions; concerns about the data.

**Figure 8:** Detailed information of the specific variables involved in the final prognostic model. **(A)** Screening of clinical variables related to OS by univariate analysis in the GC cohort. **(B)** Identification of the final variables by multivariate analysis based on the backward stepwise variable selection with the Akaike information criterion (AIC). *P* < 0.05 indicates statistical significance.

**Figure 9:** Nomogram considering glycolysis and clinical factors for prediction of the individualized survival probability of GC patients. **(A)** Development of a nomogram containing age and risk score to predict 1-, 2-, and 3-year OS. **(B–D)** Calibration plots of the nomograms in terms of the agreement between nomogram-predicted and observed 1-, 2-, and 3-year survival outcomes of the GC cohort. The 45° dashed line represents the ideal performance. The actual performances of the model are represented by the blue lines, and the figures from left to right illustrate the 1-, 2-, and 3-year results, respectively.

### Expression Levels of Seven GRGs in GC Tissues

To determine the clinical significance of the seven hub GRGs identified in GC, the expression levels of STC1, CLDN9, EFNA3, ZBTB7A, NT5E, NUP50, and CXCR4 were compared between normal gastric tissues and GC tissues using the Oncomine database (Figure 10). We found that seven GRGs were upregulated in GC tissues and downregulated in normal gastric tissues (*P* < 0.05). Furthermore, RT-qPCR was employed to verify the differential expression of genes in tumor and normal cells (Figure 11). The expression levels of STC1, CLDN9, EFNA3, ZBTB7A, NT5E, NUP50, and CXCR4 in MGC803, HGC27, and BGC823 cell lines were much higher than in GES-1 cell lines, showing no difference from the results of the Oncomine database. Therefore, we reasoned that upregulation of gene expression, mainly the expression levels of risky types (STC1, CLDN9, NT5E, and CXCR4), may produce the ultimate comprehensive effect of promoting the risk of tumorigenesis, playing an important role in poor prognosis, which needed further experimental verification.

**Figure 10:** Validation of the expression of seven GRGs at the transcriptional level between normal tissues and GC tissues by the Oncomine database. **(A)** STC1; **(B)** CLDN9; **(C)** EFNA3; **(D)** ZBTB7A; **(E)** NT5E; **(F)** NUP50; **(G)** CXCR4. *P* < 0.05 was considered to be statistically significant.

**Figure 11:** Further verification of the overexpression of seven GRGs in RT-qPCR analysis. **(A)** STC1; **(B)** CLDN9; **(C)** EFNA3; **(D)** ZBTB7A; **(E)** NT5E; **(F)** NUP50; **(G)** CXCR4. Compared to normal tissues, ns, not significant, *P < 0.05, **P < 0.01, ***P < 0.001.

The article "Seven-Gene Signature Based on Glycolysis Is Closely Related to the Prognosis and Tumor Immune Infiltration of Patients With Gastric Cancer" was retracted in 2024. Reasons: contaminated cell lines or tissues; unreliable results or conclusions; concerns about the data.

### The Expression Levels of GRGs Affected the Distribution of Immune Cell Infiltration

Different levels of immune infiltration may explain to some extent why cancer patients with the same histological type may have diverse clinical outcomes (42). Driven by the fruitful achievements in immunotherapy achieved in the field of gastric cancer treatment (9, 10), we explored the correlations of the seven GRGs and immune infiltration levels, aiming to disclose the underlying mechanism by which the seven-gene signature influenced the prognosis of gastric cancer. Violin plot analysis showed that the levels of cell infiltration, including regulatory T cells (Tregs), monocytes, M2 macrophages and resting dendritic cells, were higher in the high-risk group than in the low-risk group (*P* < 0.05), whereas the levels of follicular helper T cells (Tfh cells) and resting NK cells (*P* < 0.05) in the high-risk group were lower than in the low-risk group (Figure 12A). Clearly, the high-risk group reflected an immunosuppressive tumor microenvironment, filled with a large number of immunosuppressive cells, which coincided with the poor prognosis of the high-risk group. TIMER was then applied to assess the correlations of the expression levels of the seven GRGs with tumor purity and infiltrating levels of immune cells (Figures 12B–H). The results illustrated that the gene expression had an extremely complex and variable effect on the microscopic characterization of immune infiltration, reflecting the heterogeneity and complexity of the immune microenvironment. Intriguingly, EFNA3 (Figure 12D), ZBTB7A (Figure 12E), and NUP50 (Figure 12G), as protective types, all had a significant positive correlation with macrophage infiltration, whereas the opposite trend was presented by the results of most risk types. The correlation between genes and other immune cells is relatively weak and requires further study. These findings suggested that the seven-gene signature may play a momentous role in the formation and layout of the immune infiltration of GC.

**Figure 12:** Correlation analysis of the expression of the seven GRGs with complex immune infiltration level in GC. **(A)** Violin plot analysis comparing the distribution of various immune cell infiltrations in the high- and low-risk groups. The red group represents the high-risk group, whereas the blue group represents the low-risk group. **(B–H)** Partial correlation analysis of the expression of the seven GRGs on tumor purity and immune infiltration levels by TIMER database. **(B)** STC1; **(C)** CLDN9; **(D)** EFNA3; **(E)** ZBTB7A; **(F)** NT5E; **(G)** NUP50; **(H)** CXCR4.

The article "Seven-Gene Signature Based on Glycolysis Is Closely Related to the Prognosis and Tumor Immune Infiltration of Patients With Gastric Cancer" was retracted in 2024. Reasons: contaminated cell lines or tissues; unreliable results or conclusions; concerns about the data.

## Discussion

In recent years, increasing amounts of attention have been devoted to the research of energy metabolism, and there are inextricable links between human malignant tumors and energy metabolism. The vast majority of tumor cells are characterized by the Warburg effect, exhibiting enhanced glycolysis even under normoxic conditions, with the purpose of providing sufficient energy to support rapid biosynthesis [23,24]. Inspired by this metabolic feature, many studies on glycolysis and tumors have come into being. For instance, Yang et al. found that the miR-489-3p/SIX1 axis regulated the glycolysis level, which was important for the growth and metastasis of melanoma (43). Liu et al. conformed that lncRNA Actin Gamma 1 Pseudogene (AGPG) may be regarded as a potential biomarker and cancer therapeutic target and that inhibiting AGPG dramatically impaired glycolysis activity and cell proliferation in esophageal squamous cell carcinoma (ESCC) (44). Wang J et al. discovered that miRNA (miR)-202 expression levels were significantly lower in HCC tissues compared with normal tissue by PCR analysis, which was related to poor survival. Further, the upregulation of miR-202 expression can significantly inhibit glucose uptake, lactate production and cell proliferation of liver cancer cells (45).

However, increasing evidence has shown that single clinical factors or single gene features are susceptible to the influence of multiple factors, which makes it difficult for them to be true and reliable prognostic markers. With the swift development of high-throughput gene sequencing technology, it is possible to focus on a range of the most important functions associated with predicting patient survival, rather than extensive exploration (46). In our study, we obtained expression data and clinical materials downloaded from the TCGA database to screen out 326 GRGs. Furthermore, univariate and multivariate Cox regression analyses were performed to identify a combination of seven GRGs (STC1, CLDN9, EFNA3, ZBTB7A, NT5E, NUP50, CXCR4) with prognostic value for GC patients rather than a single gene. Subsequent survival analysis showed that the high-risk group was related to poorer prognosis, which was validated by three independent cohorts. Furthermore, we also found that the high-risk group was markedly enriched in the carcinogenic activation pathways via GSVA analysis, such as gap junction, MAPK signaling pathways, TGF beta signaling pathway, Wnt signaling pathway, which provided a more comprehensive and convincing explanation for the poor prognosis of the high-risk group. In addition, the overexpression of seven genes in tumor tissues relative to normal tissues was also confirmed in the Oncomine database and PCR analysis. Finally, risk and age were identified as independent OS-related variables, which were incorporated into the nomogram, and the results indicated that the nomogram can be regarded as a valid tool for clinical diagnosis and treatment of GC patients. These findings suggested that a seven-gene signature had powerful capacity to predict the prognosis of GC patients, which has certain guiding significance for the decision-making of clinical treatment.

The article "Seven-Gene Signature Based on Glycolysis Is Closely Related to the Prognosis and Tumor Immune Infiltration of Patients With Gastric Cancer" was retracted in 2024. Reasons: contaminated cell lines or tissues; unreliable results or conclusions; concerns about the data.

Among the seven genes, ZBTB7A, as the only gene that belongs to both protective and independent prognostic factors, has been found to be involved in the glycolysis process of tumors (47, 48). ZBTB7A, also known as POKEMON (49), FBI (50), LRF (51), and OCZF (52), is a member of the POZ/BTB and Krüppel (POK) family of transcription factors. Previous research has found that expression of ZBTB7A was associated with upregulation of glycolytic genes and lower survival in colon cancer patients, which revealed a new tumor suppressor effect of ZBTB7A in direct inhibition of glycolysis (53, 54). However, it was interesting that their results are based on the evidence that the ZBTB7A locus was frequently deleted in many human tumors, which was different from the results we verified from the Oncomine database and our PCR results, suggesting that the glycolysis of gastric cancer may have a unique pattern that requires further study. CXCR4, namely, C-X-C chemokine receptor type 4, a cognate receptor for CXCL12 (also known as stromal-derived factor 1), can mediate glycolysis programming through the CXCL12/CXCR4/mTOR signal axis, promoting the “Warburg” effect of AML cells (55). In addition, STC1 (Stanniocalcin 1) is a paracrine factor associated with inflammation and carcinogenesis that can help mesenchymal cells to protect cancer cells from apoptosis and enhance the Warburg effect (56). Similar to our results, CLDN9 (Claudin- 9) has also been identified as a glycolysis-related gene with both risk factors and independent prognostic factors in endometrial cancer and is significantly related to the prognosis of patients (17). Specifically, as far as our information goes, there is no relevant research concentrating on CLDN9, NT5E, and NUP50 in relation to tumor glycolysis. All these studies were in line with our results; however, further research is urgently acquired.

To date, much work has concentrated on tumor glycolysis. However, the biological events influenced by tumor glycolysis, especially the turbulence of their immune microenvironment, have not been well-elucidated. We found that the levels of immune cell infiltration in the high-risk group, especially immunosuppressive cells (Tregs, Macrophages M2, etc.), were significantly higher than in the low-risk group, while the low-risk group showed the opposite phenomenon, flooding the immune-positive cells (Tfh and NK cells). In other words, the high expression of GRG increased the high risk of tumor formation and led to the emergence of “cold tumors” (57), impairing the efficacy of immunity and fostering an immunosuppressive tumor microenvironment caused by high glycolysis, which was in accordance with poor prognosis. It is particularly worth mentioning that tumor-associated macrophages (TAMs) and their progenitors account for the largest proportion of medullary cells infiltrating most human solid tumors (58, 59). Macrophage polarization has become a hotspot in the research of tumor escape mechanisms in recent years and can be differentiated into classic (M1) or selective (M2) activated cells according to the changes of external conditions. Concretely speaking, M1 macrophages have a pro-inflammatory and anti-tumor effect through the expression of inducible nitric oxide synthase (iNOS), whereas the M2 macrophages (anti-inflammatory and pro-tumor) are beneficial to the growth of tumor cells and express high levels of anti-inflammatory cytokines (such as IL-10) and strong arginidase-1 (arg1) activity (60–62). Tumor glycolysis excessively converts sugar into lactic acid, which will inevitably lead to a more acidic tumor microenvironment. Studies have shown that the accumulation of lactic acid can induce macrophages to develop an inflammatory pro-tumor phenotype (63). Additionally, it has been shown that cytokines of inflammatory cells and lactic acid produced from tumor cells can form positive feedback circulation to accelerate tumor progression and invasion (64–66). Overall, we can infer that glycolysis produces ample lactic acid, which skews macrophages toward an M2-like state, providing an explanation for the close relationship between the glycolysis signature and the M2 macrophage phenotype of gastric cancer. Given this evidence, it is a fair bet that the protective types (EFNA3, ZBTB7A, NUP50) could be associated with the M1 macrophages, which have a pro-inflammatory effect, whereas the risky types (STC1, CLDN9, NT5E, CXCR4) may be relevant to the M2 macrophages, with an anti-inflammatory effect, as indicated by our results.

The article "Seven-Gene Signature Based on Glycolysis Is Closely Related to the Prognosis and Tumor Immune Infiltration of Patients With Gastric Cancer" was retracted in 2024. Reasons: contaminated cell lines or tissues; unreliable results or conclusions; concerns about the data.

Our study first identified and comprehensively analyzed the GRGs related to the prognosis of GC patients with the help of the public TCGA database. More importantly, developing a seven-gene signature to predict the outcomes of patients showed satisfactory prediction performance, but there were certain limitations in this study. However, there were certain limitations in this study. First, we verified the gene expression at the cell level *in vitro*, and the amount of cell lines was too small. *In vivo* verification at the animal level or clinical validation may be better choices. Second, there was a lack of a specific mechanism by which GRGs affected the macrophage polarization in the tumor microenvironment. In other words, given the complexity and heterogeneity of the immune microenvironment, the infiltration of immune cells should be the result of multiple factors. However, we did not consider other factors that affect the infiltration of immune cells, such as chemoresistance, different chemokines and cytokines, and the regulatory effects of different stress responsive pathways on some critical transcription factors for comprehensive analysis. It was only a preliminary study on the relationship between glycolysis level and immune cell infiltration, and the specific mechanism of action and regulatory relationship need to be further studied. Finally, some important prognostic variables, such as chemoradiotherapy and adjacent tissue inflammation extent type, were not available in the TCGA database. Hence, the impact of these variables on the nomogram is unclear.

In summary, for the first time, we identified and validated a seven-GRG signature associated with the prognosis of GC patients. The higher the risk score of GC patients, the shorter the survival period. In addition, we also found that the glycolysis of tumors was closely related to immune cell infiltration, which had a dual effect on the efficacy of immunotherapy. These results may have enlightening significance for breaking through the bottleneck of gastric cancer treatment.

## Conclusion

We formed a seven-gene signature based on the expression of STC1, CLDN9, EFNA3, ZBTB7A, NT5E, NUP50, and CXCR4 in GC, which had robust prediction capacity for patient prognosis. At the same time, this work also revealed the relationship between tumor glycolysis and tumor immune infiltration. These results introduce a novel line of thinking for the development of new targeted drugs for gastric cancer and the optimization of immunotherapy.

## Data Availability Statement

The original contributions presented in the study are included in the article/Supplementary Material, further inquiries can be directed to the corresponding author/s.

## Author Contributions

SY conceived and designed the study with CH and WL. SY and CH drafted the manuscript and analyzed the data with LC and XD. FL, QY, and LL formatted the images and the article. CZ and XL reviewed the data. YZ make a great contribution in revision progress including analysis and interpretation of data. All authors have read and approved the final published manuscript.

The article "Seven-Gene Signature Based on Glycolysis Is Closely Related to the Prognosis and Tumor Immune Infiltration of Patients With Gastric Cancer" was retracted in 2024. Reasons: contaminated cell lines or tissues; unreliable results or conclusions; concerns about the data.

## Conflict of Interest

The authors declare that the research was conducted in the absence of any commercial or financial relationships that could be construed as a potential conflict of interest.
